# Prognostic and Therapeutic Significance of Circulating Tumor Cell Phenotype Detection Based on Epithelial-Mesenchymal Transition Markers in Early and Midstage Colorectal Cancer First-Line Chemotherapy

**DOI:** 10.1155/2021/2294562

**Published:** 2021-11-03

**Authors:** Guang Lu, Zhiwen Lu, Caixia Li, Xianping Huang, Qiang Luo

**Affiliations:** People's Hospital of Luoding (Affiliated Luoding Hospital of Guangdong Medical University), No. 34 Lingyuan Road, Luoding, Yunfu, GuangDong 527200, China

## Abstract

**Purpose:**

Epithelial-mesenchymal transition (EMT) is related to the process of metastasis and challenges the detection of circulating tumor cells (CTCs) based on epithelial cell adhesion molecules. Circulating tumor cells (CTCs) have been proven to be a prognostic indicator of colorectal cancer (CRC). Although there is evidence that CTC heterogeneity based on EMT markers is associated with disease progression, no standard recommendations have been established for clinical practice. This study is aimed at evaluating the prognostic significance of dynamic CTC detection based on EMT for early and midstage colorectal cancer patients.

**Methods:**

101 patients with early to midterm CRC were admitted from January 2016 to September 2018. All patients underwent CRC radical surgery and standard chemotherapy. Patients in the postchemotherapy were able to epithelial mesenchymal transformed (EMT) CTC testing in peripheral blood using the CanPatrol™ system. Multiple CTC tests were performed according to patient's own condition and different follow-up time points. Based on patient's basic information and follow-up data, the Kaplan-Meier method was utilized to establish the progression-free survival model, and the log-rank test was utilized to compare the survival rates between the two groups.

**Result:**

Total CTC change of the patient is the best method to predict whether progression-free survival progresses in tumor patients (Area = 0.857). The second detection of total number of CTCs (*P* < 0.01) detected after chemotherapy, epithelial CTCs (*P* = 0.032), the increased total number of CTCs (*P* < 0.01), and the increased number of mesenchymal CTCs (*P* = 0.015) are significantly related with patient's poor progression-free survival.

**Conclusion:**

Analysis of the second CTC count and classification after follow-up are more related to the survival prognosis of the tumor. The joint analysis of CTC dynamic monitoring data is a good tool to judge patient's survival prognosis.

## 1. Introduction

Colorectal cancer (CRC) is one of the most common malignant tumors; the incidence rate is the third in female and the second in males globally [1]. In China, the incidence of CRC ranks the fifth in malignant tumors, and the incidence rate increases rapidly year by year [2]. With improvements of individual living standards, great changes have taken place in our lifestyles, such as increased intake of animal fat, processed meat, and red meat, reduced intake of fiber, reduced exercise, and obesity, which are considered to change composition of intestinal flora and increase the risk of colorectal cancer [3]. The 5-year survival rate of patients with CRC after surgery is 40% to 60% [4]. Treatment criteria for colorectal cancer include surgical resection and adjuvant chemotherapy. Due to the removal of colorectal cancer metastases and targeted therapy, the 5-year survival rate of patients with colorectal cancer metastases has improved in the past few years [5, 6]. Although molecular diagnosis, gene sequencing, surgical resection, and systemic adjuvant chemoradiotherapy have been successfully applied to the treatment of CRC, some patients have had liver or other organ metastasis at the time of diagnosis due to the clinical manifestations of CRC [7]. The long-term survival of patients with CRC is affected by recurrence and distant metastasis [8–10].

Circulating tumor cells (CTCs) are the general name for a variety of tumor cells that originate in the primary tumor, metastases, and other unknown minimal residual disease (MRD) sites and are released into the blood circulation [11]. There is heterogeneity among CTCs, and it is reported that abnormal activation of epithelial-mesenchymal transition (EMT) may promote tumor cell proliferation and invasion in human cancer cell lines and mouse models [12]. Using the physical and biological properties of these materials, different technologies enrich and test these materials [13]. Peripheral blood CTC number and EMT classification of various cancer patients are related to prognosis [14–16]. The number of CTCs can reflect tumor burden and detect efficacy, and it is earlier than standard imaging changes [17]. Therefore, the detection of CTC and EMT molecular typing in peripheral blood can help us to noninvasively assess the blood-borne metastasis status of cancer patients and adjust the treatment plan as soon as possible to improve its prognosis.

The purpose of this study is to study the function of single CTC count and EMT classification and multiple CTC count and EMT classification in colorectal cancer patients and to evaluate their potential diagnostic value in early and midterm CRC.

We adopt CanPatrol™ CTC typing technology [18] to analyze the number and type of circulating tumor cells in peripheral blood samples from patients with CRC, to explore the correlation between single or multiple CTC counts, EMT molecular typing, and clinical baseline of colorectal cancer, and to explore potential tools for disease progression and assessment of poor prognosis.

## 2. Materials and Methods

### 2.1. Inclusion and Exclusion Criteria

From January 2016 to September 2018, 101 patients with early to midstage colorectal cancer admitted to our hospital were included in the study. Eligible patients receive capecitabine (1000 mg/m 2 twice a day, days 1-14, every 3 weeks) plus docetaxel (75 mg/m 2 on day 1, every 3 weeks) for up to 6 cycles or until the disease progresses; the adverse event cannot be tolerated, or the patient withdraws. Each patient signed an informed consent form.

Inclusion criteria: (1) patients with pathologically diagnosed colorectal cancer; (2) patients with stage II and III clinical stage and postoperative chemotherapy.

Exclusion criteria: (1) patients with colorectal cancer have no clear pathology or cytological diagnosis; (2) clinical data and prognostic information are not perfect; (3) antitumor treatment is not acceptable.

### 2.2. CTC Detection Method

Using the CanPatrol™ assay system, 10 mL of blood was collected and transferred to a sample antiseptic tube containing ammonium chloride (Surexam Biotech, Guangzhou, China). Based on a lysis buffer via a custom connection (Surexam Biotech, Guangzhou, China), samples were incubated for 30 minutes at room temperature [18].

Red blood cells were removed by red blood cell lysis buffer, CD45+ cells were separated by 8 *μ*m diameter pore diameter, and CTCs were enriched by a membrane filter calibrated with 8 *μ*m diameter pore diameter; RNA in situ hybridization (ISH) identification based on branched DNA (bDNA) signal amplification technique characterizes CTCs and detects EMT markers [18]. According to the EMT marker, the enriched cells were classified into three subtypes of epithelial (E-) CTCs, mesenchymal (M-) CTCs, and epithelial-mesenchymal (E&M-) CTCs. Epithelial markers: epithelial cell adhesion molecule (EPCAM), cytokeratin 8(CK8), cytokeratin 18(CK18), and cytokeratin 19(CK19); mesenchymal markers: vimentin (VIM), Twist.

### 2.3. Statistical Analysis

The data was recorded in a database designed by Microsoft office Excel (Microsoft, Redmond, WA, USA), and statistical analysis was performed using IBM SPSS Statistics 25.0 software (IBM, Armonk, NY, USA). Analysis variables include gender, age, tumor size, lymph node metastasis, degree of tumor differentiation, degree of tumor invasion, tumor serological markers: carcinoembryonic antigen (CEA) and carbohydrate antigen199 (CA199), first total CTC and EMT typing CTC count, second total CTC and EMT classification CTC count, and the total CTC and EMT classification CTC count dynamically change. Perform univariate analysis and multivariate Cox regression model analysis on all variables. Survival analysis was performed by the Kaplan-Meier method to establish a progression-free survival (PFS) survival model, and the Log-rank test was utilized to compare the survival rates between groups. If the *P* value ≤ 0.05, the result is considered statistically significant.

## 3. Results

### 3.1. CTC Classification and Clinical Characteristics of Patients

This study included 101 early and midstage colorectal cancer patients; collected 101 patients' gender, age, tumor size (cm), and tumor node metastasis (TNM) staging information; and collected 35 patients with tumor differentiation, 20 patients with postoperative CEA, CA199, and other information. As shown in Figure 1, the three subtypes of CTCs in colorectal cancer patients are divided by RNA in situ hybridization. The three subtypes are E-CTCs, E&M-CTCs, and M-CTCs from left to right.

The 101 patients had a minimum age of 36 years, a maximum age of 71 years. There were 50 male cases and 51 female cases. The size of the primary tumor of patient's tumor is between 2 and 8 cm. Thirty-five patients had clinical information on tumor differentiation, 10 poorly differentiated patients, 18 moderately differentiated patients, and 7 highly differentiated patients. A total of 126 CTC tests were performed on 101 patients, and the CTC positive rate was 84.9% (107/126). The first CTC test of 101 patients after chemotherapy was in the range of 0-45/5 mL. The change range of CTCs detected by 20 patients after chemotherapy for the second time was 0-15/5 mL. The number of CTCs detected in the third and fourth times after chemotherapy was too small, and the change range was not statistically significant.

As listed in Table 1, the clinical information of colorectal cancer patients and the results of two CTC tests showed the total number of CTCs tested for the first time after chemotherapy and that E/M-CTCs and M-CTCs were significantly positively correlated with the size of the primary tumor (*P* < 0.01, *N* = 101); the second M-CTCs detected after chemotherapy were negatively correlated with the primary tumor size (*P* = 0.015, *N* = 20). The number of CTCs (*P* = 0.039, *N* = 35) and E/M-CTCs (*P* = 0.022, *N* = 35) detected for the first time after chemotherapy was inversely related to the degree of tumor differentiation. The total number of CTCs detected for the first time after chemotherapy, E/M-CTCs, and M-CTCs was also positively correlated with the degree of tumor invasion (*P* < 0.01, *N* = 101). The total number of CTCs detected for the first time (*P* = 0.046, *N* = 101), E/M-CTCs (*P* = 0.020, *N* = 101), and E-CTCs (*P* = 0.023, *N* = 101) was proportional to the number of tumor lymph nodes and the possibility of transfer.

### 3.2. Patient CTC Dynamic Detection and Patient Imaging Examination

Among the 101 patients, 81 received 1 CTC test, 17 received 2 CTC dynamic monitoring, 1 received 3 CTC dynamic monitoring, and 2 received 4 CTC dynamic monitoring. The statistics of the number of two examinations after chemotherapy in 20 patients are as follows.

Of the 20 patients, 6 had tumor progression, 10 had increased total CTCs, 2 had no change in total CTCs, 8 had a decrease in total CTCs, and 6 had tumor progression. In the increase in the total number of CTCs by 10, none of the patients with the total number of CTCs changed or decreased did not show patients with tumor progression (Figure 2(a)); there were 3 patients with elevated E-CTCs, of which 2 had tumor progression, and 1 had no tumor progression. 13 patients had the same number of E-CTCs, of which 3 had tumor progression, and 10 had no tumor progression. There were 4 patients with a decrease in the number of E-CTCs, and 1 of them had tumor progression (Figure 2(b)); there were 8 patients with elevated E/M-CTCs, of which 3 had tumor progression, and 5 had no tumor progression; 4 had no change in the number of E/M-CTCs, of which 2 had tumor progression, and 2 did not appear tumor progression. There were 8 patients with decreased E/M-CTC numbers, 1 of whom had tumor progression, and 7 others had no tumor progression (Figure 2(c)); 7 patients with increased M-CTCs, 4 of which had tumor progression, and 3 patients did not have tumor progression. 10 patients with unchanged M-CTC number, including 1 patient with tumor progression, and 9 patients without tumor progression. 3 patients with M-CTC number decline, 1 of whom tumor progression occurred, but the other 2 persons did not develop tumor progression (Figure 2(d)).

Six of the 20 patients had tumor progression, and all of them appeared in 10 of the total increase in CTCs. One of them was followed up by patient count 18 (PC18) patients. A total of 4 CTCs were tested, and the total number of CTCs continued to rise. The number of CTCs increased in PC18 patients after the second CTC test in July 2017; the third CTC test in November 2017 continued to increase the total number of CTCs. At the same time, patients underwent computed tomography (CT)examination, and patients with CT may have liver and lung metastases; in April 2018, the fourth CTC test was carried out. The total number of CTCs continued to rise. At the same time, CT examination was performed, and the patient developed liver and lung metastasis (Figure 3). Another patient, PC20, was followed up for a total of 3 CTC tests, and the number of CTCs continued to rise. In the third CTC test of this patient after chemotherapy, patient's imaging revealed multiple metastases of colorectal cancer and liver and kidney metastases. PC19 patients had a total of 4 tests during the follow-up period after chemotherapy, and the total CTCs of the patients continued to decrease to 0, and the patients did not find tumor progression.

Patient's (*N* = 20) tumor size, tumor markers CEA and CA199, and patient's total CTC (Figure 3(a)), 3E-CTC, E/M-CTC, and M-CTC dynamic changes were analyzed by receiver-operating characteristic curve (ROC), and the research results showed (Figure 3(b)) the total CTC change of the patient is the best method to predict whether PFS progresses in cancer patients (Area = 0.857), followed by the dynamic change of M-CTCs (Area = 0.685), and the other indicators are the dynamic change of E/M-CTCs (Area = 0.643), E-CTC dynamic changes (Area = 0.625), CA199 (Area = 0.601), and CEA (Area = 0.470), and the most unsuitable indicator for predicting whether PFS progresses in tumor patients is the size of the primary tumor (Area = 0.452).

### 3.3. CTCs and Tumor Progression-Free Survival

In this study, patients were followed up for PFS. Finally, 20 patients with PFS were included in the study. During the follow-up, 6 patients with early and midterm colorectal disease progressed. The median follow-up time for this study was 11 months, and the follow-up ranged from 3 months to 24 months. For age, sex, lymph node metastasis, degree of tumor differentiation, primary tumor size, total number of CTCs detected for the first time after chemotherapy (total-CTCs-1), first detection of epithelial CTCs (E-CTCs-1), first mixed CTCs test (E/M-CTCs-1), mesenchymal test (M-CTCs-1) for the first time, total CTCs test (total-CTCs-2) for the second test after chemotherapy follow-up, the second detection of epithelial CTCs (E-CTCs-2), the second detection of mixed CTCs (E/M-CTCs-2), the second detection of mesenchymal type (M-CTCs-2) and the total of two tests dynamic change of CTCs (dynamic of Total CTCs), dynamic change of epithelial CTCs (dynamic of E-CTCs), dynamic change of hybrid CTCs (dynamic of E/M-CTCs), dynamic change of mesenchymal CTCs (dynamic of M-CTCs), etc., a single clinical variable and PFS were analyzed by univariate analysis, and found tumor lymph node metastasis (*P* = 0.073). The lower degree of tumor differentiation (*P* = 0.077) and adverse PFS have a certain trend (*P* value is close to 0.05); among the results of two CTC tests after chemotherapy, the results of the first CTC test were not related to patient's PFS (Table 2). The CTC result of the second test was more related to patient's tumor progression. The results show that Total − CTCs − 2 ≥ 3/5 mL was extremely significantly related to patient's poor PFS (*P* < 0.01); E − CTCs − 2 ≥ 1/5 mL was significantly related to patients with poor PFS (*P* = 0.032 < 0.05); CTC dynamic detection and PFS univariate analysis showed that the increase in the total number of CTCs was highly correlated with patients with poor PFS (*P* < 0.01), and the number of mesenchymal CTC increased was significantly related to patients' bad PFS (*P* = 0.015 < 0.05).

Kaplan-Meier progression-free survival curve analysis (Figure 4) was performed on the univariate analysis affecting the prognosis of PFS survival. The results are as follows: the increase in the total number of CTCs is most related to the poor prognosis (*P* < 0.01). Total − CTCs − 2 ≥ 3 predicts patient's poor PFS (*P* < 0.01); the average PFS of Total − CTCs − 2 ≤ 3 and > 3 is 22.6 months and 11.07 months (Figure 4(a)); E − CTCs − 2 ≥ 1/5 mL are detected; the patient indicates poor PFS (*P* = 0.032 < 0.05); the average PFS of E − CTCs − 2 ≥ 1 and E-CTCs-2 negative are, respectively, 11.25 months and 20.41 months (Figure 4(b)). The tumor progression of the 6 patients all showed an increase in the total number of CTCs, and the PFS survival curve was significantly different (Figure 4(c)); the mean PFS of mesenchymal CTC increase and decrease was 11.33 months and 21.3 months (*P* = 0.015 < 0.05), with a significant difference (Figure 4(d)).

Subsequently, multivariate Cox regression analysis (Table 3) was performed, and the results showed that lymph node metastasis, degree of tumor, Total-CTCs -2/5 mL, E-CTCs-2/5 mL, dynamic of total CTCs, and dynamic of M-CTCs cannot be utilized as independent prognostic factors for poor PFS.

## 4. Discussion

CTCs shed from primary or secondary tumors into rare tumor cells in the peripheral blood circulation. CTCs play an important role in cancer metastasis; they are separated from the original tumor, survive in the circulation, and attach to the endothelium at the target organ, and they also invade parenchyma and finally form a tumor mass in distal site [19]. The tumor cells will be detached from the primary tumor before completely obtaining phenotype of the malignant tumor cells, or its dissemination exists in the whole process of tumor development. These early disseminated tumor cells are parallelized and evolved independently of the primary tumor. It is an important cause of postoperative recurrence and distant metastasis in patients with malignant tumors and is also an important factor leading to the death of cancer patients. Previous studies using ISET platforms or similar methods have detected CTCs undergoing EMT which helps tumor metastasis process in most patients [20, 21], which is consistent with our findings that Kaplan-Meier progression-free survival curve analysis showed that the increase in M-CTCs was predictive of poor PFS in colorectal cancer (*P* = 0.015).

Cohen et al. [22] and Gazzaniga et al. [23] reported that the detection rate of circulating tumor cells in peripheral blood circulating tumor cells of patients with colorectal cancer was significantly correlated with pathological stage. In our study, the analysis of the two CTC test results after chemotherapy found that the data of the first CTC test after chemotherapy were more related to the size of the primary tumor, lymph node metastasis, tumor differentiation, and tumor invasion. The results of Cohen and Gazzaniga and others have some consistency with ours.

Changes in the number and type of CTCs can reflect the tumor burden and detect the effect, and it is earlier than the standard imaging CT examination [17]. In breast cancer and lung cancer, there are cases reported that the number of CTC patients continues to increase, which indicates that patient's tumor progresses earlier than CT [24, 25]. In this study, the number of CTC detections of 6 patients with tumor progression increased, and the number of CTCs of patients with case number PC18 continued to increase. The CT examination corresponding to the third CTCs showed that the patients had tumor progression and liver and lung metastasis. ROC curve analysis results show that total CTC dynamic detection is the best method to predict whether PFS progresses in tumor patients (Area = 0.857).

Patients who participated in chemotherapy were regularly followed up by medical staff. The follow-up data were typical repeated measurements, including CTC testing and testing time. The advantages of multiple analysis of data to build an analytical model can dynamically monitor observer's changes over time. Analysis of the data from the two tests found that the CTC data from the second test was more relevant to the prognosis and survival of the patients. The research results show (Figure 4): the average PFS time of the second total CTCs ≤ 3/5 mL is 22.6 months, and the average PFS time of the total CTCs > 3/5 mL is 11.07 months (*P* < 0.01); the second detection test with epithelial CTCs, the patient indicates poor PFS (*P* = 0.032), and the average PFS for E − CTCs ≥ 1 and E-CTCs negative is 11.25 months and 20.41 months, respectively. The data of the second test of CTCs is different from that of the first test. The data of the first test is more related to the clinical baseline of the patient, and the data of the test during the follow-up is more related to the survival prognosis. Combined with two data analysis, the total CTC increase was significantly associated with poor PFS and significance (*P* < 0.01), the average PFS of patients with elevated M-CTCs was 11.33 months, and the PFS of decreased and unchanged patients was 21.3 months (*P* = 0.015 < 0.05). In multivariate analysis, the results of multivariate Cox regression analysis show that multiple test data cannot be adopted as independent prognostic factors for poor PFS. Hou et al. [26] showed that the emergence of M-CTCs is an independent prognostic factor for PFS in patients with advanced colorectal disease, which is inconsistent with our research results. From the correlation analysis between the data, it can be seen that the total number of circulating tumor cells detected for the first time after chemotherapy, and the CTCs that have undergone epithelial-mesenchymal transition have a certain relationship with patient's primary tumor size, tumor differentiation, tumor invasion, and lymph node metastasis. The number and type of CTCs detected for the second time during the follow-up period were not highly correlated with patient's basic clinical information of the tumor. The analysis may be due to the fact that we have detected fewer cases on multiple occasions, and this study is aimed at early and midterm colorectal patients, nonmetastatic colon cancer patients.

## 5. Conclusion

Based on the results of this study, we believe that multiple CTC tests are of great significance in CRC. The first CTC count and EMT classification after chemotherapy are more relevant to the clinical baseline of the tumor. The second CTC count and EMT classification followed by the tumor survival prognosis are more relevant. CTC dynamic monitoring data combined analysis is a good tool to judge the survival prognosis of patients. A single CTC test in colorectal cancer does not meet the clinical needs for monitoring the occurrence and development of patients' tumors. Multiple CTC monitoring at different time points is more beneficial for the evaluation of patients' tumor prognosis. Due to the limited size of our research cohort, further large-scale studies are needed to confirm our current data, and other clinical pathological records and long-term follow-up are needed to prove that multiple CTC monitoring and analysis at different time points can assess the outcome of CRC survival.

## Figures and Tables

**Figure 1:** CTC subcomponent pattern of colorectal cancer patients.

**Figure 2:** CTC dynamic changes in different subgroups of patients tested twice.

**Figure 3:** Patient's PFS progression ROC analysis chart.

**Figure 4:** Kaplan-Meier progression-free survival of colorectal cancer patients.

**Table 1:** Correlation between clinical characteristics of patients and CTCs of different subgroups.

			1-Total	1-E	1-E&M	1-M	2-Total	2-E	2-E&M	2-M
Spearman's rho	Gender	*r*	0.121	0.008	0.145	0.116	0.291	-0.050	0.294	0.267
		*P*	0.230	0.934	0.147	0.248	0.214	0.835	0.209	0.255
		*N*	101	101	101	101	20	20	20	20
	Age	*r*	0.038	-0.060	-0.036	0.170	0.118	-0.028	0.067	-0.103
		*P*	0.702	0.551	0.718	0.090	0.621	0.906	0.780	0.665
		*N*	101	101	101	101	20	20	20	20
	Size	*r*	0.508	0.083	0.475	0.390	0.078	0.013	0.363	-0.536
		*P*	0.000^∗∗^	0.411	0.000^∗∗^	0.000^∗∗^	0.745	0.956	0.116	0.015^∗^
		*N*	101	101	101	101	20	20	20	20
	Degree	*r*	-0.351	-0.100	-0.386	-0.104	0.003	-0.127	0.131	-0.071
		*P*	0.039^∗^	0.569	0.022^∗^	0.551	0.989	0.595	0.582	0.767
		*N*	35	35	35	35	20	20	20	20
	Tumor invades	*r*	0.465	0.119	0.411	0.386	0.170	-0.054	0.111	0.163
		*P*	0.000^∗∗^	0.237	0.000^∗∗^	0.000^∗∗^	0.474	0.822	0.641	0.491
		*N*	101	101	101	101	20	20	20	20
	Lymph nodes	*r*	0.199	0.226	0.232	0.093	0.203	0.364	0.065	0.120
		*P*	0.046^∗^	0.023^∗^	0.020^∗^	0.356	0.390	0.114	0.784	0.614
		*N*	101	101	101	101	20	20	20	20
	CEA	*r*	-0.216	0.076	-0.208	-0.252	-0.157	0.182	-0.145	-0.275
		*P*	0.359	0.749	0.379	0.283	0.509	0.443	0.542	0.241
		*N*	20	20	20	20	20	20	20	20
	CA199	*r*	-0.308	-0.177	-0.093	-0.264	-0.231	0.043	-0.184	-0.231
		*P*	0.186	0.455	0.695	0.260	0.328	0.857	0.437	0.328
		*N*	20	20	20	20	20	20	20	20

^∗∗^ *P* < 0.01 (2-tailed); ^∗^*P* < 0.05 (2-tailed).

**Table 2:** Single factor analysis of PFS.

Variable	PFS				
	Mean (months)	95% confidence interval		Chi-square	Log-rank *P* value
		Lower bound	Upper bound		
Age				0.038	0.845
≤55	18.21	13.725	22.685		
>55	17.75	10.770	24.730		
Gender				0.022	0.881
Male	18.51	13.342	23.683		
Female	15.06	12.016	18.095		
Lymph node metastasis				3.218	0.073
N0					
N1					
Degree of tumor				3.126	0.077
Low	14.58	9.357	19.803		
Medium/high	21.88	17.979	25.771		
Tumor size (cm)				1.126	0.289
≤4	14.58	11.447	22.286		
>4	21.88	15.988	24.699		
Total-CTCs -1/5 mL				0.177	0.674
≤3	18.735	14.011	23.459		
>3	17.500	11.682	23.318		
E-CTCs-1/5 mL				0.614	0.433
0	17.18	12.588	21.762		
≥1	21.17	16.097	26.236		
E/M-CTCs-1/5 mL				1.154	0.283
<2	10.45	8.088	12.818		
≥2	19.67	15.488	23.858		
M-CTCs-1/5 mL				0.987	0.320
0	16.66	11.923	21.399		
≥1	21.17	16.097	26.236		
Total-CTCs -2/5 mL				7.354	0.007^∗∗^
≤3	22.60	19.997	25.203		
>3	11.07	6.835	15.311		
E-CTCs-2/5 mL				4.591	0.032^∗^
0	20.41	16.802	24.017		
≥1	11.25	4.232	18.268		
E/M-CTCs-2/5 mL				2.181	0.140
<2	21.78	17.671	25.884		
≥2	15.42	10.216	20.628		
M-CTCs-2/5 mL				2.718	0.099
0	20.73	16.678	24.772		
≥1	12.75	8.317	17.183		
Dynamic of total CTCs				8.116	0.004^∗∗^
Decrease or unchanging					
Increase					
Dynamic of E-CTCs				1.659	0.198
Decrease or unchanging	19.41	15.573	23.254		
Increase	12.67	2.859	22.474		
Dynamic of E/M-CTCs				0.549	0.459
Decrease or unchanging	19.11	14.484	23.743		
Increase	12.95	8.821	17.084		
Dynamic of M-CTCs				5.937	0.015^∗^
Decrease or unchanging	21.30	17.887	24.713		
Increase	11.33	6.035	16.632		

^∗∗^ *P* < 0.01 (2-tailed); ^∗^*P* < 0.05 (2-tailed).

**Table 3:** Multivariate analysis of PFS.

	PFS				
	95% CI lower	95% CI upper	Wald	Exp(*B*)	*P* value
Lymph node metastasis	0.000	1.157∗10^197^	0.002	3.827∗10^4^	0.963
Degree of tumor	0.041	5.496	0.354	0.467	0.552
Total-CTCs -2/5 mL	0.032	16.364	0.041	0.724	0.839
E-CTCs-2/5 mL	0.120	16.697	0.077	1.418	0.782
Dynamic of total CTCs	0.000	4.770∗10^177^	0.004	2.023∗10^4^	0.952
Dynamic of M-CTCs	0.064	34.339	0.061	1.484	0.806

## Data Availability

The datasets generated and analyzed in the current study are not publicly available, but are available from the corresponding author on reasonable request.

## Additional Points

*What Does This Paper Add to the Literature?* This paper explores the prognostic assessment for colorectal cancer by dynamic changes of epithelial-mesenchymal transition typing of CTCs and provides reference for the prevention and control of cancer.
